The article "Fluidized Immobilized Carbon Catalytic Oxidation Reactor for Treating Domestic Wastewater" was published in 2023. Journal: J Environ Public Health.

# Fluidized Immobilized Carbon Catalytic Oxidation Reactor for Treating Domestic Wastewater

**DOI:** 10.1155/2023/8307957

**Published:** 2023-01-30

**Authors:** Hemadri Prasad Raju, Makendran Chandrakasu, Pachaivannan Partheeban, Baskaran Anuradha

**Affiliations:** ^1^Department of Civil Engineering, Sree Vidyanikethan Engineering College, Tirupati, Andhra Pradesh, India; ^2^Department of Civil Engineering, Wollega University, P.O. Box 395, Nekemte, Oromia Region, Ethiopia; ^3^Department of Civil Engineering, Chennai Institute of Technology, Chennai, Tamil Nadu, India

## Abstract

Treating wastewater and reusing it have become normal in the present era since the scarcity of fresh water prevails in many parts of the world. There are numerous techniques for treating domestic wastewater, and many have been explored to advance the ones already in use. This study is taken up to explore the new technology called *fluidized immobilized carbon catalytic oxidation (FICCO)*. Usually, both organic and inorganic materials are present in residential wastewater. In this study, catalyst-activated carbon produced from rice husk is added to a FICCO reactor to test the effectiveness of decreasing organic contaminants in wastewater. Six FICCO models were fabricated in this research study, and tests were conducted. The effectiveness of COD and BOD removal was investigated using six FICCO models with activated carbon made from rice husk as a catalyst and presented in this paper. The FICCO reactor was also used to treat organic contaminants such as surfactants, starch, oil, and protein with rice husk as activated carbon as a catalyst. Organic pollutants used the FICCO reactor; COD removal varied from 75.6% to 92.4%, BOD removal ranged from 74.9% to 89.5% at the optimum contact time, and catalyst rice husk-activated carbon application. The optimum catalyst dosage was 12 g per 620 ml of wastewater, which is the capacity of each reactor and a substantial reduction in sludge.

## 1. Introduction

Domestic wastewater (sewage), which typically contains 40 to 60% dissolved materials, 5 to 10% colloidal materials, and balance suspended materials, contributes significantly to pollution. The need for wastewater treatment in India has grown due to the country's expanding industries and population. This sector will use the most treated wastewater for production and home purposes. Over many years, coagulation, flocculation, and oxidation techniques have been developed to remove organic matter (expressed as BOD and COD) from wastewater produced by domestic and industrial processes. Even though the time needed for treatment is shorter, those procedures are expensive because they require the addition of chemicals and trained employees. Additionally, post-pH adjustment and chemical sludge treatment are necessary before disposal.

### 1.1. Literature Survey on Catalyst Hydrocarbon

According to several studies [1–8], granular activated carbon may remove a variety of organic compounds from water. Many contaminants are stable organic compounds that are not completely removed by waste treatment, either chemically or biologically. They frequently withstand the stream's natural self-purification process. More so than others, some organic contaminants can be absorbed. Organic solvents such as trichloroethylene and aromatic solvents like toluene are adsorbable because of their low solubility in water. Alcohols and aldehydes, on the other hand, are poorly absorbed by the body [9]. Activated carbon granules or air stripping are frequently used to remove volatile organic compounds (VOCs) such as low molecular weight-chlorinated solvents and aromatics. Granular-activated carbon can reduce organic pollutants to undetectable ones [10].

To reduce organic pollutants in wastewater, it is suggested that a fluidized immobilized carbon catalytic oxidation (FICCO) reactor cell with low sludge generation be studied and evaluated. A complicated environment develops as the contaminated water stream passes over a thin layer of activated carbon, forming a mass transfer zone. Contaminants are absorbed by the surface of mesoporous-activated carbon (MAC), which is used for this purpose. Immobilized cell treatment technology enables productivity growth by lowering the output of surplus sludge. The purpose of this study is to demonstrate the ability of the FICCO reactor system to remove dissolved organics such as BOD and COD from the residential sewage effluent in Adyar, Chennai.

The COD and BOD removal efficiency of the FICCO reactor was improved while adjusting the catalyst loading and time to determine the most efficient removal of organic pollutants. If rice husk carbon is employed, the investment cost of a sewage treatment plant would be greatly reduced. There would be a significant reduction in the operational cost of electrical energy use [11]. The catalytic functionalization oxidation reactor (CFOR), heterogeneous-activated carbon Fenton catalytic oxidation (HAFCO), Fenton-activated carbon catalytic oxidation (FACCO), and fluidized immobilized cell carbon oxidation were some of the methods used by the authors. Combined catalytic reactors destroyed phenol with a 96.7% efficiency, 100% of sulphide without releasing it into the environment, 95.3% of COD, and 99.2% of BOD.

### 1.2. Literature Survey on Fluidized Immobilized Carbon Catalytic Oxidation Technology

The removal of dissolved organics from home wastewater by an integrated oxidation process was proved by experimental tests using UV-visible and Fourier-transform infrared spectroscopy [12]. The most recent studies on biochar and hydrochar manufacturing, characterisation, and prospective applications have been examined. The effects of reaction temperature, feedstock types, and thermochemical conversion modes were contrasted with biochar. There was also discussion on the benefits and difficulties of encouraging the use of biochar in energy and the environment, such as adsorbents, catalytic precursors, soil amendment, anaerobic digestion and composting, and electrochemical energy storage materials. The authors also discussed the future directions for biochar research and development [13].

To produce various silicon-based chemicals and active carbon, rice husks (RHs) are processed [14] and evaluated critically. The impacts of various process parameters on the pyrolysis stage, the effect of physical, chemical, and thermal treatments, activating conditions, and the mechanisms of activated carbon consolidation were all discovered as alternative processing methods. An acidic stream is necessary to neutralise the effluent during biological wastewater treatment when pH is neutral. As a result, a very deadly gas called hydrogen sulphide is released. This work removed COD from wastewater and sulphide in lime sulphide liquor using the heterogeneous peroxide oxidation (HPO) method. Wastewater's sulphide was catalytically oxidised to sulphate by cleaving protein molecules, and the ammonia level was raised by roughly 78.05% [15].

The authors discussed the fluidized bed reactor's uses in wastewater treatment [16] and highlighted the crucial design and operational factors that affect the reactor's performance. Fluidized bed reactors for liquid-solid and gas-liquid-solid processes, all effective methods for treating wastewater, were examined, as was the applicability of these processes in advanced oxidation, biological, and adsorption processes. A wastewater treatment system that is both energy- and money-efficient is necessary for the industry to adopt cleaner manufacturing. There were some recommendations for potential research topics at the end of the review. The properties of the sorbent texture and the amount removed do not appear to be directly related. The order in which phenol absorption rises is 2-CP, P, Cr 4-NP 2, 4-DNP 2, 4-DCP.

The authors [17] talked about various ways to make activated carbon (AC) from rice husk (RH) precursors as well as its uses. Applications for the environment, catalysis, and energy have all been noted. Future chances for development and research were also analyzed. Overall, it was found that RH-derived AC holds much promise for various uses that can be further researched on a practical scale, i.e., for prospective industrial services. In a review of recent studies on activated conversions of emerging contaminants, metal-free techniques have been highlighted as one of the most significant advancements. At the end, cutting-edge coupling procedures and some prospects were presented [18].

The methods for removing (or degrading) emerging trace organic contaminants are described in this paper. Alkylphenols and their polyethoxylated derivatives, which are thought to interact with the wildlife's hormonal system, were the subject of the study, which concentrated on one type of endocrine disruptor. A fascinating technique for treating alkylphenol is photocatalytic oxidation since it can achieve entire mineralisation [19]. This study demonstrates the high efficiency of the wet air oxidation method for converting the majority of contaminants to carbon dioxide. It has been shown that energy net generation typically occurs throughout a continuous process. This research is considered the first step for creating a large-scale wet air oxidation unit [20].

Worldwide production of maize husk and rice husk (MS/RH) makes them desirable and economically advantageous feedstocks for large-scale biochar manufacturing for environmental remediation. As a result, the authors [21] thoroughly describe the preparation, characterisation, and environmental remediation of pure and composite MS/RH biochar. Other wastewater treatment research studies that have used an experimental laboratory setting include those by Ahmad et al. [22], Bond et al. [23], Zhang et al. [13], Watanabe [24], Snowden et al. [25], Liu et al. [26], Liu et al. [27], Kennedy et al. [28], Hasler et al. [29], and Van Haandel et al. [30–32]. As demonstrated by the preceding method, FICCO and rice husk wastewater treatment is a novel technique, which is why this study is being conducted.

### 1.3. Objectives of the Study

It is learnt from the above literature survey on these lines that there was a scope for exploration of a new technique to improve the treatment efficiency. In this study, triangle-shaped sheets with different angles were introduced at the top for sufficient catalyst retention in the reactor to study its effects on removal efficiencies of COD and BOD from domestic wastewater. This research's main objective is to design and test experimentally to find COD and BOD removal efficiency at the optimum contact time and catalyst dosage. Furthermore, the removal of COD and BOD caused by individual organic pollutants such as surfactants, starch, oil, and proteins separately by artificial addition was explored.

## 2. Materials and Methods

### 2.1. Collection of Domestic Wastewater (Sewage) and Rice Husk

The sewage treatment facility (STP), Adyar, Chennai, provided wastewater, and Table 1 lists its basic characteristics. To create activated carbon, rice husk, a raw material acquired from the agricultural sector, was extensively cleaned with water to eliminate dust. Later, a 600 *μ*m sieve was used to filter dry samples.

### 2.2. Preparation of Rice Husk-Activated Carbon

Porous carbon was produced via precarbonisation and chemical activation. The rice husk was heated to 400°C for four hours during the precarbonisation stage and then allowed to cool naturally to ambient temperature. As a result of this procedure, precarbonised carbon was produced (PCC). Precarbonised carbon was stimulated by subsequent chemical activation. 250 g of an aqueous solution containing 85% H_3_PO_4_ was mixed by weight with 50 g of precarbonised carbon during the chemical activation process. The precarbonised carbon to chemical triggering agent ratio was determined at 4.2 pH. At 85°C for 4 hours, precarbonised carbon and the chemical activator were well mixed. Precarbonised carbon slurry was mixed and vacuum-dried for 24 hours at 110°C. The samples were then heated to 700°C for 1 hour at a 100 mL/min flow rate in a vertical cylindrical furnace with regular air. Activated carbon was cooled, repeatedly rinsed with hot water until the pH was neutral, and then washed with cold water to remove any phosphorus compounds that could have remained. To create the finished product, 110°C drying was applied to the washed samples.

### 2.3. FICCO Reactor Models

Fluidized immobilized carbon catalytic oxidation (FICCO) reactors, which have a 9 cm square plan and a 12 cm height, were made from acrylic sheets. Triangles were fixed at the top to ensure smooth flow and efficient operation of the fluidized system for wastewater treatment. These reactors were constructed with 620 mL working volumes and 740 mL reactor volumes with an aeration provision. The fluid bed was kept in place, and air circulation was made possible by using the air distribution system.  Figure 1 depicts the models that were created. A typical 3D view of the outline diagram of the FICCO model with a triangle slope at the top and side by using the settling tank is shown in Figure 2. Each reactor provided with a different angled triangle slope at the top is shown in Figures 3(a)–3(f).

### 2.4. Operation of FICCO Reactors

During the conduction of experiments with FICCO reactors, initial COD and BOD concentrations are maintained constant. At the same time, the optimum contact time and carbon dosage are used for the performance studies on the effectiveness of COD and BOD removal.

Wastewater enters the reactor from the bottom and overflows when it reaches the triangle's top surface, spilling into the adjacent tank. Triangles are barriers to keeping activated carbon in the reactor for a predetermined time by changing the flow rate. To obtain greater efficiency in removing COD and BOD, activated carbon must slide down and remain in the reactor for a long period on the smooth surface provided by the slope of the triangles at the top. The air distribution system is designed to maintain the fluid bed while allowing air to circulate for oxidation.

## 3. Results and Discussion

Experimental research made use of FICCO reactor models (Figures 3(a)–3(f)). The catalyst's optimum dosage and contact time for domestic wastewater were obtained to continue the study and validate the findings.

### 3.1. Performance Studies Using FICCO Reactors

Initially, performance studies using FICCO reactors were conducted for the removal efficiency of contaminants without the addition of activated carbon. Raw sewage and FICCO-treated wastewater were analyzed for characteristics including pH, sulphates, chlorides, COD, BOD, total suspended solids, and oil and grease, as shown in Table 1.

As presented in Table 1, without catalyst-activated carbon, BOD and COD removal efficiencies are 53.65 and 53.74, respectively. The performance of this will be improved with the use of catalyst. Initially, the optimum dose of the catalyst prepared using rice husks and the optimum contact time required for removal of BOD and COD were experimentally observed, and the same was used in the research work to explore various options such as different triangle shapes provided at the top of FICCO models 3A to 3F.

### 3.2. Optimum Dose of Rice Husk-Activated Carbon

It is observed from Table 1 that without an activated carbon catalyst, the average BOD and COD reduction efficiency through this experiment is only about 53.65% and 53.74%, respectively. Thus, the significance of catalyst loading is elucidated with experimental studies. The effect of catalyst mass loading on COD during the catalytic oxidation of domestic wastewater is shown in Figure 4.

The average percentage of COD reduced rose from 22% to around 90% as catalyst loading was increased from 1 to 12 g per 620 ml while the contact time was kept constant at 150 minutes. There was no increase in percentage COD removal as catalyst mass loading was increased from 12 to 15 g per 620 ml. Under current operating conditions, a catalyst concentration of 12 g per 620 ml can thus be deemed optimal.

### 3.3. Optimum Contact Time

COD and BOD removal studies were conducted with an optimum 12 g per 620 ml dosage to determine the optimum contact time.  Figure 5 illustrates the proportion of COD and BOD removed with and without the catalyst as a function of time. The ratio of COD removed with and without motivation grew steeply for the first 3 hours and then gradually for the next 2 hours, reaching 57% and 92% from 54% to 90%, which is meagre. The proportion of BOD removed was similar to that of BOD released at about 44% and 82% in 3 hours and reached nearly 46% and 84%, respectively, in the next 2 hours, which is a meagre change. Hence, 3 hours is considered the optimum contact time. So the optimum contact time is considered for further studies as 180 minutes, since the removal efficiency is not significant after 3 hours of the contact time.

### 3.4. Performance of the FICCO Reactor with Catalyst-Activated Carbon Made from Rice Husks

Each FICCO reactor is equipped with a triangle slope, as shown in Figures 3(a)to 3(f). Initially, the constant flow was applied to FICCO reactors, with a continuous concentration of COD and BOD to all *A* to *F* reactors. Then, aeration was started with an immobilized cell reactor system with appropriate aeration. At an optimum hydraulic retention time (HRT) of 3 hours, an inlet flow containing a predetermined concentration of COD and BOD was continually supplied into the reactor and analyzed for inlet and outlet results.  Table 2 lists the COD and BOD removal efficiency of each of the six reactors conducted with the predetermined optimum dose of activated carbon and the optimum contact time. The enhanced average percentage removal of COD and BOD compared to reactors without the catalyst and triangle slopes confirmed the robust working of the FICCO reactor with those arrangements. The results improved from around 53% to about 84% on average.

It is observed from Table 2 that the maximum and minimum removal efficiencies of COD are 92.4% and 75.6%, respectively. The maximum and minimum BOD removal efficiencies are 89.5% and 74.9%, respectively. The average of all six FICCO reactors' efficiency in COD removal is 84.13%, and in BOD, it is 80.71%. This is higher than in the results obtained without the catalyst, which are presented in Table 1. In Table 1, COD and BOD removal efficiencies without the addition of catalyst-activated carbon are 53.74% and 53.65%, respectively. With the addition of catalyst-activated carbon made from the rice husk, the removal efficiency of COD increased by about 30.39% and that of BOD by approximately 27.06%, which is a substantial amount of removal. Another observation is that the FICCO reactor shown in Figure 3(c) with a 45° triangle-shaped slope has shown higher efficiency than the other slope angles of triangles. This can be attributed to the angle at which catalyst-activated carbon retains sufficient time before leaving the settling tank, which facilitates a slightly higher adsorption rate.

## 4. Performance of the FICCO Reactor for the Removal of Specific Organic Pollutants

Further studies were explored using the FICCO reactor, especially “3C” type, which has a 45° slope triangle shape at the top of the reactor, giving the maximum efficiency in removing COD and BOD. Individual organic pollutants, such as surfactants, starch, oil, and proteins, were added to water, and the performance of the FICCO reactor was studied. The results of studies are presented in Sections 4.1to 4.4, and also, sludge characteristics are also analyzed and presented in Section 4.5.

### 4.1. Performance of the FICCO Reactor for Removal of Surfactants

The effect of anionic surfactant concentration on the performance of the FICCO reactor was investigated. Wastewater at a surfactant concentration of 23.8 mg/L was introduced into the reactor and operated for a week at an optimum catalyst dosage of 12 mg per 620 ml and a contact time of 3 hours, and every day samples from the input and outlet were collected and analyzed. The results are shown in Figure 6. The maximum removal efficiencies of COD and BOD were found to be 82.7% and 81.5%, respectively, which is shown in the graph (Figure 4). The average COD and BOD removal efficiencies were 76.37% and 74.97%, respectively. The average outlet concentration of surfactants was 4.8 mg/L. Anionic surfactants are readily biodegradable under aerobic conditions as opposed to anaerobic conditions, at which they are unlikely to be degraded.

### 4.2. Performance of the FICCO Reactor for Removal of Starch

The effect on the performance of the FICCO reactor was explored with the addition of starch. The reactor was operated with the same optimum catalyst dose of 12 g per 620 ml and at an optimum contact time of 3 hours. Experiments were conducted for about a week, and daily samples of the input and output were collected and analyzed whose results are shown in Figure 7. The initial starch content was 32.1 mg/L in wastewater. The average outlet concentration of starch after treatment was 5 mg/L. The maximum COD and BOD removal efficiencies were found to be 88.1% and 87.7%, respectively. The average COD and BOD removal efficiencies were 76% and 74.2%, respectively. This clearly shows that the aeration process with a catalyst in this reactor can reduce the starch content substantially within a short period.

### 4.3. Performance of the FICCO Reactor for Removal of Oil

The performance of the FICCO reactor was studied with the concentration of adding oil in addition to surfactants and starch separately. The reactor was operated with the same optimum catalyst dose of 12 g per 620 ml and at an optimum contact time of 3 hours. Experiments were conducted for about a week, and daily samples of the input and output were collected and analyzed whose results are shown in Figure 8. The wastewater's influent concentration of oil was 45 mg/L. The average effluent concentration of oil using the FICCO reactor was found to be 6 mg/L. The maximum COD and BOD removal efficiencies were 85.2% and 84.1%, respectively. The average COD and BOD removal efficiencies were calculated to be 75.7% and 72.64%, respectively.

### 4.4. Performance of the FICCO Reactor for the Removal of Protein

The performance of the FICCO reactor was studied with the concentration of adding protein in addition to surfactants, starch, and oil separately. The reactor was operated with the same optimum catalyst dose of 12 g per 620 ml and at an optimum contact time of 3 hours. Experiments were conducted for about a week, and daily input and output samples were collected and analyzed, as shown in Figure 9. The wastewater's influent concentration of protein was 33.7 mg/L. The average effluent protein concentration using the FICCO reactor was 4.27 mg/L. The maximum COD and BOD removal efficiencies were 85.5% and 77.1%, respectively, for protein contamination. The average COD and BOD removal efficiencies were calculated to be 72.65% and 70.76%, respectively.

### 4.5. Sludge Characteristics of Treated Organic Pollutants

The sludge production and its characteristics for all the given four conditions of adding a surfactant, starch, oil, and protein are presented in Table 3. After 7 days of continuous running, sludge was collected using the reactor, and the experiments on sludge characterisation were studied. It is observed from Table 3 that sludge produced per 35 litres of organic pollutant surfactant, starch, oil, and protein is 720 ml, 730 ml, 643 ml, and 1210 ml, respectively. It is a meagre amount compared to the volume of wastewater treated. Hence, disposal costs, including transportation costs, reduce substantially.

## 5. Conclusions

Using a fluidized immobilized carbon catalytic oxidation reactor with aeration and activated carbon made from rice husks effectively lowers the quantity of organic contaminants found in domestic wastewater. With carbon-based rice husk-activated carbon, the average removal efficiencies of COD and BOD content from domestic sewage were observed to be 84.13% and 80.71%, respectively, which have improved substantially from 53.74% to 53.65%, respectively. Almost 30% improvement is seen from the results after adding catalyst-activated carbon made from rice husks. Sludge generation was also reduced substantially; only 60% of typical sewage treatment plants in the FICCO treatment facility produced sludge output. Hence, the carbon-based rice husk significantly reduces the construction expenditure and operational costs of the sewage treatment facility.

With a 3-hour contact period and an appropriate dosage of 12 g per 620 ml of the effluent, the FICCO reactor gives a substantial 30% more efficiency in removing COD and BOD when compared without catalyst-activated carbon. In addition to providing the catalyst with the proper dose and contact duration, equipping the reactor with a 45° slope triangle makes it simple to keep catalyst-activated carbon for adequate time to use it for organic contamination adsorption effectively.

Wastewater after FICCO reactor treatment can be let into an algal pond, where it might undergo additional treatment through an algal cycle before being released into the environment or reused. Finally, it is concluded that with rice husk-based catalyst-activated carbon and the FICCO reactor model, the overall removal efficiency of COD and BOD is substantial. Hence, this can be employed for treating domestic wastewater cost effectively and efficiently where space constraints exist since this type of treatment requires less space and takes only 3 hours of contact.

## Figures and Tables

**Figure 1:** FICCO reactor (models *A* through *F*).

**Figure 2:** A typical 3D view outline diagram of the FICCO reactor model.

**Figure 3:** (a)–(f) Shapes of the triangles with different slopes provided at the top of the FICCO reactor. (a) Triangle with 40°. (b) Triangle with 40°. (c) Triangle with 45°. (d) Triangle with 50°. (e) Triangle with 50°. (f) Triangle with 55°.

**Figure 4:** Percentage removal of COD as a function of catalyst loading.

**Figure 5:** Percentage removal of COD and BOD as a function of time.

**Figure 6:** COD and BOD removal % with the addition of surfactants.

**Figure 7:** COD and BOD removal % with the addition of starch.

**Figure 8:** COD and BOD removal % with the addition of oil.

**Figure 9:** COD and BOD removal % with the addition of protein.

**Table 1:** Physicochemical parameters of raw and FICCO-treated wastewater without the addition of catalyst-activated carbon.

S. no	Parameters	Raw wastewater	FICCO treated	Removal efficiency (%)
1	pH	7.6 ± 0.6	8.2 ± 0.2	—
2	BOD	171.1 ± 51.7	79.3 ± 5.2	53.65
3	COD	514.7 ± 154.6	238.1 ± 16.5	53.74
4	Total suspended solids	187.1 ± 60	82.6 ± 9.6	55.85
5	Nitrogen	50.2 ± 21.6	31.1 ± 5.8	38.05
6	Sulphate	36.1 ± 10.3	16.3 ± 5.9	54.84
7	Chlorides	40 ± 6	13.2 ± 3.7	67.00
8	Oil and grease	60 ± 8.9	16 ± 1.8	73.33

*Note*. All parameters are expressed in mg/L except pH.

**Table 2:** COD and BOD removal efficiency of different FICCO reactors *A* to *F*.

FICCO reactors *A* to *F*	COD % removal	BOD % removal
*A*	75.6	74.9
*B*	84.2	79.2
*C*	92.4	89.5
*D*	86.7	82.8
*E*	85.6	81.4
*F*	80.3	76.5

Average	84.13	80.71

**Table 3:** Sludge characteristics.

Parameters	Surfactant	Starch	Oil	Protein
Wet sludge weight (g/ml)	3.551	3.9356	1.1401	1.2837
Dry sludge weight (g/ml)	0.5795	1.0527	0.4384	0.7186
Sludge volume (ml/L)	0.72	0.73	0.643	1.21
The volume of compressed sludge (ml/L)	0.0936	0.369	0.257	0.164
Fixed solids (g/L)	0.048	0.057	0.036	0.004
Specific weight (g/ml)	3.5	1.3118	1.14	1.28
Sludge density (g/ml)	0.0599	0.368	0.215	0.0269
Filter sludge compressed (g/ml)	0.7	0.85	0.5384	0.1186

## Data Availability

The data used to support the findings of this study are available from the author upon request.
